The article "Metronomic combination chemotherapy using everolimus and etoposide for the treatment of non‐Hodgkin lymphoma" was published in 2019. Journal: Cancer Med.

# Metronomic combination chemotherapy using everolimus and etoposide for the treatment of non‐Hodgkin lymphoma

**DOI:** 10.1002/cam4.2364

**Published:** 2019-06-20

**Authors:** Ke Wu, Xiao‐Qing Sun, Cai‐Qin Wang, Tian‐Xiao Gao, Peng Sun, Yu Wang, Wen‐Qi Jiang, Zhi‐Ming Li, Jia‐Jia Huang

**Affiliations:** ^1^ Department of Medical Oncology, Sun Yat‐sen University Cancer Center, State Key Laboratory of Oncology in South China Collaborative Innovation Center for Cancer Medicine Guangzhou China

**Keywords:** metronomic combination chemotherapy, NHL, RAD001, VP‐16

## Abstract

Patients with Non‐Hodgkin lymphoma (NHL) treated by conventional chemotherapeutic drugs usually require a long recovery period. However, metronomic combination chemotherapy (MCC) enhances therapeutic efficacy and decreases side effects in the treatment of NHL. In this study, we tested and compared the effects of metronomic chemotherapy (MC) using podophyllotoxin derivative etoposide (VP‐16) alone and that of MCC using both VP‐16 and everolimus (RAD001) in the treatment of NHL. Two types of NHL cells, OCI‐LY‐10 and SU‐DHL‐6, were employed for the experiments. Cell proliferation, apoptosis, and cell senescence were measured to test the effects of drugs in each experiment. In addition, the influences of MC and MCC on the cell cycle and autophagy pathway were evaluated to study the functional mechanisms behind their effects. Finally, we conducted analyses of the growth inhibitory effect and synergistic activity for different MCC. The results showed that MC using low‐dose VP‐16 alone demonstrated strong treatment effects in terms of inducing apoptosis, cell senescence, and reducing tumor cell proliferation, and this treatment also led to changes of the cell cycle. Compared with MC, MCC using VP‐16 and RAD001 together demonstrated even stronger treatment effects, with both the cell cycle and autophagy‐related proteins being affected. Considering the synergistic activity, our results showed the MCC of VP‐16 48 hours + RAD001 24 hours is the optimal method for treating NHL.

## 1 INTRODUCTION

Non‐Hodgkin lymphoma (NHL) encompasses a diverse group of malignancies that are distinguished by specific cancer cell characteristics in accordance with each disease subtype associated with different treatments. Cytotoxic chemotherapy remains the frontline treatment for NHL. This treatment mode requires chemotherapeutic agents in every cycle reaching the maximum tolerated dose (MTD), from which a long recovery period is needed.^1^ Moreover, the off‐therapy interval provides a good opportunity for tumor cells to acquire drug resistance and regrow, leading to treatment failure.^2^

To minimize these problems, a new treatment modality of drug administration called “metronomic chemotherapy” (MC) has been proposed. MC exerts an anti‐proliferative effect with relatively mild and short‐lived toxic effects. MC is administered via a low‐dose and high‐density approach, with no extended drug‐free breaks. Researchers reported that MC outperforms MTD strategies in tumor cells with different growth rates,^2^ and that MC provides better treatment for chemo‐resistant tumors, which has been supported by multiple preclinical model studies.^2^, ^3^, ^4^

Meanwhile, combination chemotherapy (CC) may further augment the accumulation of anti‐tumor effects, improving the therapeutic efficacy. Indeed, CC has shown great potential in NHL. For example, Kummar reported that veliparib in combination with metronomic cyclophosphamide was well tolerated.^5^ In addition, Zeng reported, in 2016, that MCC with prednisone, etoposide, and cyclophosphamide resulted in higher ORR(objective response rate) and DCR (disease control rate) in patients with relapsed or refractory non‐Hodgkin lymphoma.^6^ Therefore, developing more effective combination MC strategies is important.

The article "Metronomic combination chemotherapy using everolimus and etoposide for the treatment of non‐Hodgkin lymphoma" was published in 2019. Journal: Cancer Med.

Among the diverse combination strategies available, chemotherapy combined with targeted treatment has been demonstrated to be superior to combinations of conventional chemotherapeutic agents. However, for non‐Hodgkin lymphoma, therapeutic toxify and effects remains much more to explore. Deregulation of the mTOR pathway has been proven to be a factor contributing to various types of cancer,^7^ including lymphoma.^8^ In addition, researchers reported that the mammalian target of rapamycin (mTOR) pathway governs growth signals associated with diverse processes, including senescence,^9^ autophagy,^10^ and apoptosis.^11^ RAD001 is an inhibitor of the mammalian target of mTOR.^4^ Previous studies demonstrated that RAD001 alone had anti‐proliferative effects in various malignancies, including renal cancer, breast cancer, non‐small cell lung cancer, and pancreatic neuroendocrine tumors.^12^, ^13^, ^14^, ^15^ Moreover, studies showed that mTOR inhibitors in combination with other traditional chemotherapeutic agents (cyclophosphamide, doxorubicin, vincristine，prednisone) presented better efficacy in treating NHL.^16^, ^17^, ^18^

The podophyllotoxin derivative etoposide (VP‐16) is known to be one of the most effective chemotherapeutic drugs. Substantial research has confirmed its role in the treatment of a number of malignancies including lymphoma. VP‐16 works by inducing DNA strand breaks through a topo II‐mediated mechanism.^19^

However, to date, no study has been conducted to test the effect of administering MC using low‐dose VP‐16 versus metronomic combination chemotherapy (MCC) using both VP‐16 and RAD001 in the treatment of NHL. By reason of DNA damage inducing autophagy, even apoptosis.^20^ Therefore, we assumed that a synergistic effect on NHL occured upon the administration of MCC with VP‐16 and RAD001.

The article "Metronomic combination chemotherapy using everolimus and etoposide for the treatment of non‐Hodgkin lymphoma" was published in 2019. Journal: Cancer Med.

## 2 MATERIALS AND METHODS

In this study, we tested and compared the effect of administering MCs using VP‐16 alone and that of MCCs using combinations of VP‐16 and RAD001 in the treatment of NHL. Specifically, we first used the MTS assay to determine the 30% inhibitory concentration (IC_30_) of VP‐16 and RAD001 for the treatment of two different NHL cells, OCI‐LY‐10 and SU‐DHL‐6. The IC_30_ values were used for in all the experiments conducted here. Next, we measured the cell proliferation, apoptosis, and cell senescence under each treatment to evaluate the effects of the administered agents. In addition, we measured the influence of the MCs and MCCs on the cell cycle and autophagy pathway to study the functional mechanisms behind the effects of the two drugs. We also conducted analyses evaluating the growth inhibitory effect and synergistic activity of different MCCs.

### 2.1 Cells and drugs

OCI‐LY‐10 and SU‐DHL‐6 cells were chosen for the experiment. The agents RAD001 and VP‐16 were purchased from Selleck Company.

### 2.2 Dosage determination

MTS assays were used to determine the 30% inhibitory concentrations (IC_30_) and 50% inhibitory concentrations (IC_50_) of VP16 and RAD001 in the treatment of the two different cells; then, the lower (IC_50_) were used in the MC and MCC experiments.

### 2.3 MC using VP‐16 alone

The two different cells were separated into five groups: (a) control group: treated with no drugs; (b) 24 hours group: treated with VP‐16 for 24 hours; (c) 96 hours group: treated with VP‐16 for 96 hours; (d) 24 + 48 hours group: treated with VP‐16 for 24 hours and then cultured without drug for 48 hours; and (e) 96 + 48 hours group: treated with VP‐16 for 96 hours and then cultured without drug for 48 hours. Here, the dosages of VP‐16 were determined as described above, for the two different cell types. Note that the 24 hours and 24 + 48 hours groups were only used in the determination of IC_30_ and IC_50_.

After treatment, the following experiments were performed for each group to analyze the treatment effect of MCs using VP‐16 alone and to study its functional mechanisms: (a) measurement of proliferation of tumor cells by the MTS assay; (b) determination of apoptosis using TUNEL detection and annexin‐V PI detection; (c) evaluation of cell senescence using the *β*‐gal staining assay; (d) counting of cells in different phases of the cell cycle by flow cytometry and BD Accuri C6; and (e) determination of the expression levels of proteins involved in the autophagy pathway using western blotting. The first three experiments were used to assess the direct effect of treatment with MC on NHL tumor cells, while experiments (d) and (e) were performed to study the functional mechanisms behind this.

The article "Metronomic combination chemotherapy using everolimus and etoposide for the treatment of non‐Hodgkin lymphoma" was published in 2019. Journal: Cancer Med.

### 2.4 MCC using VP‐16 and RAD001

The same measurements as performed for the MCs were also applied in the MCC experiments, but with different groups: (a) 96 + 48 hours group: cultured without drugs, used as a control group; (b) R + V 48 hours group: cultured with both VP‐16 and RAD001 for 48 hours; (c) R48 hours + V24 hours group: cultured with RAD001 for 48 hours and then with VP‐16 for 24 hours; (d) V48 hours + R24 hours group: cultured with VP‐16 for 48 hours and then with RAD001 for 24 hours; (e) V48 hours group: cultured with VP‐16 for 48 hours; and (f) R48 hours group: cultured with RAD001 for 48 hours.

### 2.5 Analytical method

Statistical analyses were performed using an isobologram analysis to measure the VP‐16 and RAD001 combination index (CI). This method was performed as reported previously.^18^

## 3 RESULTS

### 3.1 Dosage determination for VP‐16 and RAD001

For both MCs and MCCs, we first used MTS assays to determine the dosage of the two drugs to be used. The obtained results are presented in Table 1. Considering the low‐dosage requirement for MC and MCC, we chose IC_30V = _0.08 µmol/L and IC_30R = _0.29 µmol/L for OCI‐LY‐10 cells, corresponding to the treatments using VP‐16 and RAD001, respectively. For SU‐DHL‐6 cells, we chose IC_30V = _1.98 µmol/L and IC_30R = _0.26 µmol/L. The determined dosages were applied for all the following ACs and ACCs in which the two drugs were used.

**Table 1:** The IC_30_ and IC_50_ Values of OCI‐LY10 and SU‐DHL‐6 cells after treatment using VP‐16 or RAD001 alone

Drug	Group	IC_30_ (µmol/L)	IC_50_ (µmol/L)
For VP‐16	OCI‐LY‐10 treated by VP‐16 for 24 h	2.12	7.30
	OCI‐LY‐10 treated by VP‐16 for 96 h	**0.08**	0.14
	SU‐DHL‐6 treated by VP‐16 for 24 h	14.84	34.14
	SU‐DHL‐6 treated by VP‐16 for 96 h	**1.98**	4.10
For RAD001	OCI‐LY10 treated with RAD001 for 48 h	**0.29**	0.6
	SU‐DHL‐6 treated with RAD001 for 48 h	**0.26**	0.5

Both of the two groups are *P* < 0.05 (in bold).

### 3.2 Effect of MC using VP‐16 alone on cell proliferation

For the three groups (control group, 96 hours group, and 96 + 48 hours group), we measured the optical density (OD) values of each group and present the results in Figure 1A,B. The results showed that the 96 hours groups for both cell types demonstrated significantly low OD values, indicating that low‐dose MC possesses strong anti‐proliferative effects. Notably, the 96 + 48 hours group demonstrated a higher OD value than the 96 hours group, suggesting that tumor cell proliferation partially recovered after cessation of the continuous treatment using VP‐16.

The article "Metronomic combination chemotherapy using everolimus and etoposide for the treatment of non‐Hodgkin lymphoma" was published in 2019. Journal: Cancer Med.

**Figure 1:** Effect of MC using VP‐16 alone on cell proliferation. (A, B) The OD values measured in the MTS assay. Both OCI‐LY‐10 and SU‐DHL‐6 cells were divided into three groups: 1) control group: treated with no drugs; 2) 96 h group: treated with VP‐16 for 96 h; and 3) 96 + 48 h group: treated with VP‐16 for 96 h and then cultured with no drug for another 48 h. (C, D) The distribution of cell number of OCI‐LY‐10 and SU‐DHL‐6 under different MCs using VP‐16. G_1_ is the period of cell growth before the DNA is duplicated; S is the period when DNA is duplicating; G_2_ and M is the period after DNA duplication and the period of the mitotic phase

In addition, we measured the numbers of cells in different phases of the cell cycle, as shown in Figure 1C,D. The results showed that there were changes in the cell cycle in terms of the relative numbers of cells in G_1_ and S phases but not in interphase (G_2_) and the mitotic (M) phase. The percentage of cells in the S phase increased, indicating that cell cycle arrest associated with VP‐16 might be caused by the induction of DNA damage, further influencing cell proliferation. These results imply that the anti‐proliferative activities of MC using VP‐16 are superior to those in conventional chemotherapy.

### 3.3 Influence of MC with VP‐16 on cell senescence and autophagy pathway

Our *β*‐gal staining assay results also suggested that VP‐16 can induce cell senescence (Figure 2A,B). In addition, the 96 + 48 hours groups for both cell types demonstrated optimal effects in terms of the observed aging of cells. It was reported that cell senescence can activate the autophagy pathway.^21^, ^22^ Therefore, we also tested the relative quantity of a set of proteins associated with the autophagy pathway using western blotting, including Atg5, Beclin 1 (BECN1), mTOR, LC3B, cl Caspase3 (CASP3), and GAPDH. These genes are also regulators of apoptosis and senescence,^23^, ^24^ as shown in Figure 2C,D. The results showed that MC with VP‐16 influenced the quantity of all these genes except GAPDH. Specifically, with the MCs, the expression levels of Atg5, Beclin1, LC3B, and cleaved (cl) Caspase3 increased while that of mTOR decreased. The increase of Atg5, Beclin 1, LC3B and the decrease of mTOR indicated the enhancement of autophagy, while the decrease of mTOR and the increase of cl caspase3 indicated the increase of apoptosis. Moreover, the variations were most significant in the 96 + 48 hours group, supporting the assertion that the effect of VP‐16 is maintained for a period after the treatment. This may help to explain how MC with VP‐16 influences tumor cell proliferation.

The article "Metronomic combination chemotherapy using everolimus and etoposide for the treatment of non‐Hodgkin lymphoma" was published in 2019. Journal: Cancer Med.

**Figure 2:** Influence of MC with VP‐16 on cell senescence and autophagy pathway. (A, B) The senescence effects of VP‐16 on OCI‐LY‐10 and SU‐DHL‐6 cells. (C, D) Western blot analysis of proteins within the autophagy pathway in OCI‐LY‐10 and SU‐DHL‐6 cells

### 3.4 Influence of MC with VP‐16 on apoptosis

We expected significant changes in terms of the absolute number of total cells after VP‐16 treatment. As shown in Figure 3A,D, apoptosis increased significantly in both the 96 hours group and the 96 + 48 hours group for both cell types. Moreover, much more significant apoptosis was observed in the 96 + 48 hours group. This indicates that the effect of VP‐16 is maintained for a certain period (ie, 48 hours) after treatment, which is consistent with the results of western blotting and β‐gal staining assay. The results from annexin‐V PI detection (Figure 3A,D) and TUNEL detection (Figure 3E,F) confirmed the above observations and suggested the effectiveness of MC with VP‐16 in inducing apoptosis.

**Figure 3:** Influence of MC with VP‐16 on cell apoptosis. (A–D) The apoptosis of OCI‐LY‐10 and SU‐DHL‐6 cells under different MCs with VP‐16 detected by Annexin‐V PI. In (A) and (B), the groups showing significant differences in the statistical comparisons are marked as follows: *compared with control (1st column); ^#^compared with 96 h group (2nd column). Significant *P*‐value: 0.05, using Tukey's multiple comparison tests. (E, F) The apoptosis of OCI‐LY‐10 and SU‐DHL‐6 cells under different MCs with VP‐16 detected by TUNEL

### 3.5 Influence of MCCs using VP‐16 and RAD001 on cell proliferation

As shown in Figure 4A,B, all groups with treatments presented relatively low OD values compared with the control group (96 + 48 hours), especially the three MCC groups (R24 hours + V48 hours, R48 hours + V24 hours, and V48 hours + R48 hours). The results suggested that MCCs could produce improved treatment effects compared to VP‐16 or RAD001 used alone. Next, we identified changes in the distribution of cell number in each group, as shown in Figure 4C,D. In particular, in the R48 hours + V24 hours group (OCI,8.27%;SU‐DHL‐6,9.95%) and the V48 hours + R24 hours (OCI‐LY‐10,3.48%;SU‐DHL‐6,4.8%) group, we identified decreased percentages of cells in the G_2_/M stage, indicating that the cell cycle was inhibited under the treatment in these two groups.

**Figure 4:** Influence of MCCs using VP‐16 and RAD001 on cell proliferation. (A, B) OD values of OCI‐LY‐10 and SU‐DHL‐6 cells under different MCCs. Cell proliferation was assessed using the MTS assay. (C, D) The changes of cell cycle associated with MCCs using VP‐16 and RAD001 on NHL cells

The article "Metronomic combination chemotherapy using everolimus and etoposide for the treatment of non‐Hodgkin lymphoma" was published in 2019. Journal: Cancer Med.

### 3.6 Influence of MCCs on cell senescence

Besides apoptosis, our results from the *β*‐gal staining assay also suggested that the three MCCs can exert stronger effects of inducing cell senescence compared to monotherapy (Figure 5A,B). As shown in Figure 5C,D, all of the treatments affected the expression levels of the tested autophagy pathway proteins, which are also regulators of apoptosis (mTOR, cl caspase3), and senescence (Atg5, Beclin 1), which in turn influenced the proliferation of the cells. After drugs administrated, Atg5, Beclin 1 significantly increased indicated the enhancement of cell autophagy and the increase of senescence phenotypes cells. Down‐regulated of mTOR implied the increase of cell apoptosis. In summary, as shown in Figure 5C,D, treatment with VP‐16 48 hours combined with RAD001 24 hours, RAD001 48 hours combined with VP‐16 24 hours and RAD001 48 hours combined with VP‐16 48 hours induced the most significant cell autophagy, senescence phenotypes, and apoptosis. The effect of treatment with VP‐16 or RAD001 alone was much weaker than that with VP‐16 and RAD001 combination. Notably, the three MCCs exerted stronger effects than V48 and R48, especially on the proteins Atg5, Beclin 1, and mTOR. This helps to explain the observation that more intense apoptosis was identified among these three groups.

**Figure 5:** Influence of MCCs on cell senescence. (A, B) The effects of different MCCs on the senescence of OCI‐LY‐10 cells by β‐gal staining assay. (C, D) The changes in expression level of the proteins within the autophagy pathway in OCI‐LY‐10 and SU‐DHL‐6 cells under MCCs

### 3.7 Influence of MCCs on apoptosis

The experiment showed that all three groups of MCCs demonstrated significantly increased apoptosis compared with the control group or with the use of VP‐16 or RAD001 48 hours alone. Moreover, the R 48 hours + V 48 hours group demonstrated the best effects for both cell types (Figure 6A,B). The results from Annexin‐V PI detection (Figure 6C,D) and TUNEL detection (Figure 6E,F) were consistent with the above observations. especially when R + V are used simultaneously, could be more effective for treating NHL.

**Figure 6:** Influence of MCCs on cell apoptosis. The groups showed significant different in the statistical comparison were marker with ^'*#&$%'^: *compared with control (1st column); ^#^compared with RAD001 group (2nd column); ^&^compared with Vp‐16 group (3rd column); ^$^compared with R + V 48 group (4th column); ^%^compared with V48 h + R24 h group (5th column). Significant p‐value: 0.05, using Tukey's multiple comparison tests.

The article "Metronomic combination chemotherapy using everolimus and etoposide for the treatment of non‐Hodgkin lymphoma" was published in 2019. Journal: Cancer Med.

### 3.8 Growth inhibition of different MCCs

Here, we compared the inhibitory effects on cancer cell growth of different MCCs at different dosages. As shown in Figure 7A,B, with increasing dosage, cell growth inhibition increased. Meanwhile, the three MCCs demonstrated greater inhibitory effects on both OCI‐LY10 and SU‐DHL‐6 cells than the use of VP‐16 or RAD001 alone. We compared the synergistic activity of different MCCs using a combination index (CI) measured by isobologram analysis. Efficacy was determined using CalcuSyn software to analyze the CI (Figure 7C,D). For OCI‐LY10 cells, synergistic activities with CI < 1 were observed for all MCCs with a different effective dose (ED). However, for SU‐DHL‐6 cells, ED_50_ of R + V and R48 + V24 hours demonstrated an antagonistic effect (CI > 1), while V48 hours + R24 hours groups exhibited additive interactions (CI = 1). In summary, we recommend the V48 hours + R24 hours as the most optimal strategies.

**Figure 7:** Growth inhibition of different MCCs. (A, B) Growth inhibition effect of different MCCs for OCI‐LY10 and SU‐DHL‐6 cells. Absorbance values were normalized to be within [0%, 100%], using the values from untreated cells. Compared with the use of single agent alone, the groups with significantly increased growth inhibition effects (*P* < 0.05) are marked with an asterisk, as evaluated using Tukey's multiple comparison test. (C, D) Synergistic activity of different MCCs on OCI‐LY10 and SU‐DHL‐6 cells

## 4 DISCUSSION

Chemotherapy plays an important role in the comprehensive treatment of cancer. However, conventional chemotherapy with MTD has limitations associated with its side effects, including the need for a long period of recovery between treatment cycles.^25^ Against this background, MC has demonstrated multiple advantages compared with conventional chemotherapy, including minimal side effects, a shorter drug‐recovery period, and less drug resistance.^26^

Initially, MC was reported to mainly target vascular endothelial cells, rather than tumor cells themselves. In this way, the acquisition of drug resistance can be reversed or avoided. However, the mechanisms of its anti‐tumor activity also include effects on immune responses and direct effects against cells that establish tumors.^27^ In recent years, as PD‐1, CTLA4, and other immune checkpoint inhibitors have played increasingly important roles in anti‐tumor therapies, immune responses have become a focus of increasingly serious interest. The immunostimulatory effects of MC include the induction of immunogenic cancer cell death, enhancement of dendritic cells’ antigen presentation, regulatory T cells’ preferential depletion, and enhancement of the cytotoxic activity of immune effector cells. These multiple targets of MC confirm its efficacy for refractory and relapsed malignancy.^28^

The article "Metronomic combination chemotherapy using everolimus and etoposide for the treatment of non‐Hodgkin lymphoma" was published in 2019. Journal: Cancer Med.

The drugs selected for use in MC strategies always have the features of being orally administered, hypotoxicity, and low economic toxicity. As noted earlier, MC combined with targeted therapy increased anti‐tumor efficacy. The most commonly reported combination is MC and the antiangiogenic agent bevacizumab in ovarian carcinoma.^29^

VP‐16 was previously demonstrated to be effective in NHL.^30^ We thus simulated clinical drug treatment using long‐term and continuous exposure of NHL cells in a culture to a low concentration of VP‐16 in MC. The results showed that the in vitro anti‐proliferative activity of low‐dose VP‐16 in NHL cells was accompanied by increased tumor cell apoptosis and senescence, which supports previous reports describing that MC could induce better treatment effects.^5^ The results also showed that the highest tumor cell apoptosis and senescence under MCs using VP‐16 alone occurred in the 96 + 48 hours group rather than the 96 hours group (Figure 2 and Figure 3), which is consistent with the changes in autophagy‐related proteins (Figure 2). These findings indicated that the effect of VP‐16 is maintained within a certain period (eg, 48 hours) after the cessation of treatment. However, the cell proliferation of the 96 + 48 hours group was higher than that of the 96 hours h group, indicating that the effect of VP‐16 decreased after the cessation of drug administration (Figure 1). This indicates that the continual administration of VP‐16 is necessary for improved efficacy.

In our studies, we also observed changes of the NHL cells in terms of the cell cycle (Figure 2). Specifically, there was an increase in the number of cells in the S phase and a decrease of those in the G_1_ phase for both cell types. Our observations are consistent with the finding that VP‐16’s target topoisomerase II is significantly expressed only in dividing cells during selected mitotic phases of the cell cycle.^31^ Topo II cleaves DNA and generates transient double‐strand breaks in the DNA.^32^ The anti‐tumor drug VP‐16 can stabilize the enzyme‐cleaved DNA complexes, which then damages DNA integrity. DNA damage activates the DNA repair pathway.^33^ In this way, the number of cells in the S phase increases. Furthermore, we noted that the MC with VP‐16 affected the expression levels of autophagy related proteins, which are also regulators of apoptosis and cell senescence (Figure 3). This is because, when the damage is severe, cells cannot repair themselves, which activates the autophagy pathway.^34^ Our findings also reveal that MC with VP‐16 exerted a much stronger effect on these regulators, which is consistent with better efficacy as described previously.^35^

The article "Metronomic combination chemotherapy using everolimus and etoposide for the treatment of non‐Hodgkin lymphoma" was published in 2019. Journal: Cancer Med.

Our results of MCC experiments using both VP‐16 and RAD001 showed that, compared with the use of one drug alone, MCCs could produce even better anti‐proliferative effects in terms of apoptosis and cell senescence (Figures 5 and 6). The improved anti‐tumor effect may arise from the fact that the MCCs with both VP‐16 and RAD001 could induce G_1_ and G_2_ cell cycle arrest (Figure 4) and influence the proteins in the autophagy pathway as well (Figure 5), which affect the proliferation of the tumor cell group. RAD001 is an inhibitor of mammalian target of rapamycin (mTOR),^36^ which is an atypical serine and threonine kinase that is found in two different complexes: mTOR complex 1 (mTORC1) and mTOR complex 2 (mTORC2). mTOR is the core component of these two complexes. However, RAD001 is only an mTORC1 inhibitor.^37^ mTORC1 is a major growth regulator that senses different nutritional and environmental factors in combination, including growth factors, energy levels, cellular stress, and amino acids. Combined with these signals, it promotes cell growth by phosphorylating substrates to enhance anabolism (such as mRNA translation and lipid synthesis) or to limit catabolism (such as autophagy).^37^ Inhibition of the mTOR pathway enhances cell cycle arrest, inhibits proliferation, and promotes the autophagy of damaged tumor cells and even their apoptosis.^38^ The possibility exists that this is associated with the synergistic effect of VP‐16 and RAD001. Although the three MCCs (R + V48 hours, R48 hours + V24 hours, and V48 hours + R24 hours groups) demonstrated similar in vitro anti‐proliferative activity, the V48 hours + R24 hours group outperformed the R + V48 hours and R48 hours + V24 hours groups in the synergistic activity analysis, with CI ≤ 1 for both types of NHL cells of all different EDs (Figure 7).^39^ Therefore, we recommend the V48 hours + R24 hours MCC as the best treatment approach.

In summary, the results of this study suggest that MC using VP‐16 alone is effective for the treatment of NHL and that the MCC method combining VP‐16 and RAD001 could lead to even better results. Our results suggest that the metronomic combination of anti‐tumor drugs with different functional mechanisms may lead to the improved treatment of NHL.

## CONFLICTS OF INTEREST

The authors declare that they have no conflicts of interest.

## Data Availability

The authenticity of this article has been validated by ploading the key raw data onto the Research Data Deposit public platform (www.researchdata.org.cn).
